The article "Ultrasound Radiomics-Guided Iliac Fascia Block on Postoperative Cognitive Dysfunction in Elderly Patients Undergoing Hip Surgery" was published in 2022. Journal: Comput Math Methods Med.

# Ultrasound Radiomics-Guided Iliac Fascia Block on Postoperative Cognitive Dysfunction in Elderly Patients Undergoing Hip Surgery

**DOI:** 10.1155/2022/2492667

**Published:** 2022-05-17

**Authors:** Jun Zha, Jinping Ni, Shuo Chen, Haijun Feng, Tuanjie Che, Shigang Qiao

**Affiliations:** ^1^Faculty of Anesthesiology, Affiliated Suzhou Science & Technology Town Hospital of Nanjing Medical University, Suzhou, Jiangsu 215153, China; ^2^Department of Anesthesiology, Suzhou Kowloon Hospital, Shanghai Jiaotong University School of Medicine, Suzhou, Jiangsu 215028, China; ^3^Laboratory of Precision Medicine and Translational Medicine, Affiliated Suzhou Science and Technology Town Hospital of Nanjing Medical University, Suzhou 215153, China; ^4^Gansu Key Laboratory of Functional Genomics and Molecular Diagnosis, Lanzhou 730000, China

## Abstract

**Objective:**

Elderly patients with hip surgery are prone to postoperative cognitive dysfunction (POCD), leading to health management difficulties. This study is aimed at investigating the effect of ultrasound radiomics-guided iliac fascia block on POCD.

**Methods:**

A total of 67 cases of patients who had undergone hip joint surgery were divided into a training set (*n* = 47) and a validation set (radiomics-guided group, *n* = 20). The patients were intervened with ultrasound radiomics-guided iliac fascia block, and the maximum relevance minimum redundancy sifts out the image omics features obtained from 2D ultrasound images of patients. Another 20 patients undergone general anesthesia served as control. The incidence of POCD, the total amount of fentanyl, the visual analogue score (VAS) at different time points, and the levels of CRP and NSE in plasma were compared between the two groups.

**Results:**

The AUC on the training and validation sets were higher than 0.940. The incidence of POCD in the radiomics-guided and general anesthesia group was 5% and 30%, respectively (*P* = 0.037). Compared with the general anesthesia group, the dosage of fentanyl in the radiomics-guided was lower, the VAS score at 6 h, 1 d, and 2 d after operation was smaller, and the levels of CRP and NSE were lower (all *P* < 0.05).

**Conclusions:**

For elderly patients with hip surgery, the ultrasound radiomics-guided iliac fascia block can reduce the incidence of POCD and improve the effect of nerve block.

## 1. Introduction

The postoperative cognitive dysfunction (POCD) often occurs in elderly patients; it refers to a series of neurological complication after surgery [1–3]. Early intervention can reduce the incidence of POCD and minimize the degree of brain injury [4, 5]. Therefore, intervention in the influencing factors of POCD is an effective measure to reduce the occurrence of POCD.

The article "Ultrasound Radiomics-Guided Iliac Fascia Block on Postoperative Cognitive Dysfunction in Elderly Patients Undergoing Hip Surgery" was published in 2022. Journal: Comput Math Methods Med.

In addition to old age, pain is also considered a high risk factor for POCD [6–9]. The mechanism of central inflammatory response also plays an essential role [10]. Patients with hip disease not only have severe pain before the operation but also suffer from pain interference after the operation [11–14], resulting in abnormal difficulty in health management. Therefore, appropriate preoperative and postoperative analgesia may be helpful for the control of POCD.

In the surgical treatment of hip joint lesions, some studies have shown that iliac fascia block can play a better analgesic effect and reduce postoperative complications [15–19]. However, it is not clear whether POCD can be affected. The radiomics features are of great value in diagnosing clinical diseases and evaluating treatment response [20–22]. In recent years, the clinical application has gradually increased. In this study, based on iliac fascia block ultrasound radiomics-guided, we tried to reduce the impact of surgery on COPD in addition to reducing pain.

## 2. Materials and Methods

### 2.1. General Information

All the participants were patients in Suzhou Science and Technology Town Hospital and Suzhou Kowloon Hospital for elective surgery in patients with hip disease. The research design was approved by the ethics committee of our hospital, and the operation plan was informed consent of patients and their families.

Inclusive criteria are as follows: hip joint surgery patients, normal nerve function can cooperate with treatment, and age ≥ 60 years. Exclusion criteria are as follows: patients with a history of mental or neurological diseases, patients with abnormal visual or auditory function, patients with severe organ abnormalities, and patients with missing clinical and follow-up data or voluntarily applying to withdraw from the study.

Finally, 87 patients were enrolled in the study, including 55 males and 32 females. Among then, 67 cases were divided into a training set (*n* = 47) and a validation set (radiomics-guided group, *n* = 20) according to the 10-fold crossover method. Another 20 patients undergone general anesthesia served as the control group.

### 2.2. Anesthesia Method

The general anesthesia group was given sufentanil 0.5 *μ*g/kg, propofol medium/long chain fat emulsion 2.5 mg/kg, rocuronium 0.8 mg/kg intravenous anesthesia induction, after the human pump propofol 6 mg/kg/h, and 0.8 MAC sevoflurane to maintain anesthesia.

The radiomics-guided group was blocked in the iliac fascia space: supine, the affected side of the limb slightly extended outward, conventional disinfection spread sterile towel, the Sonosite S-nerve color Doppler was used. After the probe was placed vertically at the position of anterior superior iliac spine, it was rotated about 20° clockwise and then moved slowly to the middle and outer 1/3 of the anterior superior iliac spine and pubic symphysis. The probe was adjusted to determine the structure of the iliac fascia space. When the needle tip penetrates below the iliac fascia, inject 30 mL of 0.25% ropivacaine hydrochloride after no blood is drawn back, pay attention to the diffusion of local anesthetic to the head, and keep the needle route within the visual range to prevent the needle from entering the abdominal cavity too deep.

The article "Ultrasound Radiomics-Guided Iliac Fascia Block on Postoperative Cognitive Dysfunction in Elderly Patients Undergoing Hip Surgery" was published in 2022. Journal: Comput Math Methods Med.

### 2.3. Postoperative Analgesia

Patients in both sets were given patient-controlled intravenous analgesia. Fentanyl (20 *μ*g/kg) was dissolved in 100 mL 0.9% sodium chloride solution. The injection speed was controlled at 2 mL/h and locked for 15 min. The single self-control volume was 0.5 mL.

### 2.4. Image Preprocessing and Region of Interest Segmentation

Image preprocessing can be divided into two steps: image gray balance and image noise reduction. Histogram equalization reduces feature differences caused by image gain differences between patients. To reduce the influence of image noise on image omics feature extraction, median filtering is applied to image denoising.

Image segmentation was performed manually by an ultrasound physician. Region of interest (ROI) was plotted on the maximum cross-section of the injected ultrasound image of each patient. The complete structural range of iliac fascia was plotted by adjusting the spatial structure position. The segmented images were finally validated by an ultrasound physician with 5 years of experience. The specific flow chart for image preprocessing and region of interest segmentation is shown in Figure 1.

### 2.5. Radiomics Analysis

The deep learning model in this research is generated by the Deep Red AI Toolbox. Firstly, the image omics features of the region of interest are extracted from the preprocessed images. Then, the extracted features are normalized to make the data normalized and conform to the standard normal distribution. The transformation function is as follows:

(1) $$\begin{array}{c} x^{*}=\frac{\left(\chi -\bar{x}\right)}{\sigma }. \end{array}$$

In addition, the maximum relevance minimum redundancy (mRMR) and the least absolute shrinkage and selection operation (LASSO) algorithm sift out the image omics features obtained from 2D ultrasound images of patients and establish the image omics score.

The mRMR algorithm is a feature selection method that maximizes the correlation between feature variables and targets and minimizes the correlation between features. More mutual information is used to measure the feature redundancy and the correlation between categories, and information entropy and information difference are used to select the optimal feature subset.

(2) $$\begin{array}{c} \text{I}\left(x,y\right)=\iint P\left(x,y\right)\log\frac{P\left(x,y\right)}{P\left(x\right)P\left(y\right)}dxdy. \end{array}$$

In the formula, *x* and *y* are given two random variables, *P*(*x*, *y*) is the joint probability distribution function of *x* and *y*, and *P*(*x*) and *P*(*y*) are probability distributions of *x* and *y*, respectively.

The article "Ultrasound Radiomics-Guided Iliac Fascia Block on Postoperative Cognitive Dysfunction in Elderly Patients Undergoing Hip Surgery" was published in 2022. Journal: Comput Math Methods Med.

To find the feature subset *S* containing *m* features, the following formula can be used to calculate its correlation:

(3) $$\begin{array}{c} \max D\left(S,c\right);D=\frac{1}{\left|S\right|}\underset{x_{i}\in S}{\sum }I\left(x_{i};c\right). \end{array}$$

A subset with *m* features may not be the best subset of features, and when two features are highly interdependent and one of them is removed, the class discrimination of the two will not change much.

The selection of variables is mainly based on the LASSO algorithm proposed by Tibshirani et al. in 1996 [23]. The loss function is as follows:

(4) $$\begin{array}{c} \min_{\beta }\overset{N}{\underset{n=1}{\sum }}{\left(y^{n}-\overset{m}{\underset{P=1}{\sum }}\beta_{p}x_{p}^{n}\right)}^{2}+\lambda \overset{m}{\underset{P=1}{\sum }}\left|\beta_{p}\right|, \end{array}$$

where *y*^*n*^ is the category label of the *N*th sample and *N* is the number of samples. *λ* is the regularization parameter, which controls the sparsity of the model.

### 2.6. Evaluation Index

The incidence of POCD, the operation time, and the total amount of fentanyl were recorded.

The visual analogue score (VAS) was used to evaluate patients' pain before the operation, 20 minutes after the puncture, 6 hours after the operation, and 1, 2, and 3 days after the operation.

The right jugular vein blood was collected before operation and at 6 h, 1 d, 2 d, and 3 d after operation. The levels of CRP (C-reactive protein) and neuron specific enolase (NSE) in plasma were detected by enzyme-linked immunosorbent assay (ELISA). Taking into account the influence of intraoperative bleeding and transfusion, the postoperative results were recorded, and corrected values were used, and the calculation was as follows:

(5) $$\begin{array}{c} \text{Corrected value}=\text{measured value}\times \frac{\text{HCT before anesthesia}}{\text{actual HCT}}. \end{array}$$

### 2.7. Statistical Methods

The SPSS 21.0 software was used for statistical analysis. The area under the receiver operating characteristic (ROC) curve was used to evaluate the effectiveness of the model. The count data were described by frequency and constituent ratio, and the comparison between the radiomics-guided and general anesthesia groups was performed by chi-square test. Quantitative data are expressed as the mean ± standard deviation. Shapiro–Wilk tests were performed to determine the normality of the data distributions. If the measurement data conform to the normal distribution, use *t*-test to compare between above two groups.

The article "Ultrasound Radiomics-Guided Iliac Fascia Block on Postoperative Cognitive Dysfunction in Elderly Patients Undergoing Hip Surgery" was published in 2022. Journal: Comput Math Methods Med.

## 3. Results

### 3.1. Diagnostic Efficacy of Radiomics Models

The selected models were evaluated, and the AUC of the model on the training set was 0.942 (95% CI 0.890-0.994), and the AUC of the model on the validation set was 0.941 (95% CI 0.885-0.996). The ROC curve is shown in Figure 2.

### 3.2. Comparison of General Information and Surgical Features

The basic information of patients is shown in Table 1. There was no significant difference in gender, age, and BMI between the radiomics-guided and general anesthesia groups (*P* > 0.05). All patients successfully completed hip surgery; postoperative showed promising results (Figures 3 and 4). The operation time of the radiomics-guided group was 96.4 ± 26.3 min, while that of general anesthesia group was 97.7 ± 31.2 min. There was no significant difference between the two groups (*P* > 0.05). The incidence of POCD in the radiomics-guided group was significantly lower than that in the general anesthesia group (5% vs. 30%, *χ*^2^ = 4.329, *P* = 0.037). The dosage of fentanyl in the radiomics-guided group was 411.5 ± 47.2 *μ*g, and that in the general anesthesia group was 738.7 ± 82.4 *μ*g, and the dosage of fentanyl in the radiomics-guided group was significantly less than that in the general anesthesia group (*P* < 0.05).

### 3.3. VAS Scores at Each Time Point

The VAS scores in the radiomics-guided and general anesthesia groups are shown in Figure 5. Compared with the general anesthesia group, the radiomics-guided group decreased significantly 20 minutes after puncture and 6 hours, 1 day, and 2 days after operation.

### 3.4. Serological Indexes at Each Time Point

The detailed comparison of CRP and NSE between the radiomics-guided and general anesthesia groups before and after the operation is shown in Table 2. Compared with that before operation, CRP and NSE increased significantly at each time point after operation, especially in the general anesthesia group.

## 4. Discussion

### 4.1. Analysis of POCD in Elderly Patients with Hip Surgery

The cognitive dysfunction is a common complication after hip arthroplasty. The incidence rate of POCD increases with age. The clinical incidence rate of elderly patients is 40% to 50% [24–26]. Anxiety, cognitive impairment, memory impairment, attention deficit, language, and social skill decline are common clinical manifestations, which seriously affect the quality of life of patients after. However, some scholars pointed out that surgical stress, operation time, physiological characteristics, anesthetic methods, extracorporeal circulation, anesthesia mode, residual anesthetic, and postoperative pain may be closely related to this complication [6–9]. Elderly patients still need general anesthesia because of their long-term special body position intolerance, difficulty in puncture in spinal canal, and use of anticoagulants and other factors, which may lead to postoperative cognitive dysfunction.

The article "Ultrasound Radiomics-Guided Iliac Fascia Block on Postoperative Cognitive Dysfunction in Elderly Patients Undergoing Hip Surgery" was published in 2022. Journal: Comput Math Methods Med.

### 4.2. Advantages of Combined General Anesthesia and Iliac Fascia Block

Peripheral nerve block is often used as an important supplement and auxiliary means of general anesthesia [15–17]. The anesthetic effect is clear, which can shorten the recovery time, reduce the dosage of general anesthetic, and effectively reduce the incidence rate of related complications. Among various regional block techniques, iliac fascia space block is a simple and easy to master technique. Its mechanism is to inject local anesthetics into the space between the iliac fascia and the iliac muscle. Then, the femoral nerve and lateral femoral cutaneous nerve between them were blocked assisted by ultrasound-guided operation. This technology is used to treat the pain of patients with hip diseases, with rapid onset and exact effect. Some studies scored the pain of patients admitted to the emergency department [15, 27, 28]. It was found that the preoperative score was high, and the pain was not well controlled. However, immediate iliac fascia space block could effectively control the preoperative pain.

### 4.3. Comparison of Diagnostic Efficacy of Radiomics Models

The results showed that the AUC of ultrasonic image radiomics in the training set (AUC: 0.942, 95% CI 0.890-0.994) and the validation set (AUC: 0.941, 95% CI 0.885-0.996) is similar. It is proved that the ultrasonic image radiomics has great efficiency for the successful puncture.

### 4.4. Comparison of POCD Characteristics

The dosage of fentanyl in the radiomics-guided group was significantly lower than that in the general anesthesia group. The VAS score in the radiomics-guided group was significantly lower than that in the general anesthesia group at 6 h, 1 d, and 2 d after operation. In addition, the incidence of POCD in the radiomics-guided group (5%) was significantly lower than that in the general anesthesia group (30%). All these results indicated that the ultrasound radiomics-guided iliac fascia block can reduce the incidence of POCD after hip operation in elderly patients.

The article "Ultrasound Radiomics-Guided Iliac Fascia Block on Postoperative Cognitive Dysfunction in Elderly Patients Undergoing Hip Surgery" was published in 2022. Journal: Comput Math Methods Med.

### 4.5. Comparison of CRP and NSE Levels

Some studies have shown that the central nervous system damage in patients with serum CRP and other inflammatory factors [29]. The CRP is an important cytokine with extensive biological activity in human body, which plays an important role in the central neuropathy progression. NSE is an enzyme widely existing in neurons, and its level changes are closely related to the degree of brain injury and prognosis of patients. Some studies have pointed out that inflammatory reaction and chronic oxidative stress reaction may lead to the synthesis and secretion of NSE [30, 31]. When it accumulates in the brain, it may lead to memory loss and progressive cognitive impairment. In this study, the CRP and NSE levels in both groups increased in a short period of time, indicating that proinflammatory factors are related to cognitive function. Compared with the general anesthesia group, the dosage of fentanyl in the radiomics-guided was lower, and the levels of CRP and NSE after operation were also lower. The results indicate that the ultrasound radiomics-guided iliac fascia block can reduce the use of general anesthesia drugs, reduce the release of inflammatory factors after and during operation, and improve postoperative cognitive function.

## 5. Conclusion

In conclusion, for elderly patients with hip surgery, the ultrasound radiomics-guided iliac fascia block can reduce the incidence of POCD and improve the effect of nerve block. However, the number of samples in this study is small, which needs to be further studied. The patients included in this study were insufficient and came from the same center. In addition, sufficient specimen is essential in ensuring the machine learning model's efficiency.

## Figures and Tables

**Figure 1:** Flow chart of image preprocessing and region of interest segmentation.

**Figure 2:** The ROC curve of ultrasound radiomics models: (a) training set; (b) validation set.

**Figure 3:** Typical case of internal fixation from a patient with hip fracture: (a) before operation; (b) after operation.

**Figure 4:** Typical case of hip replacement: (a) before operation; (b) after operation.

**Figure 5:** The VAS scores at each time point.

**Table 1:** General information between the radiomics-guided and general anesthesia groups.

Groups	*n*	Gender		Age (years)	BMI (kg/m^2^)
		Male	Female		
Radiomics-guided		14	6	69.6 ± 7.1	22.4 ± 2.7
Control		12	8	67.2 ± 5.8	21.9 ± 2.3
*x* ^2^/*t* value		0.440		1.170	0.630
*P* value		0.507		0.249	0.532

**Table 2:** Serological indexes at each time point.

Index	Radiomics-guided group	General anesthesia group	*t* value	*P* vlaue
CRP (mg/L)				
Before operation	3.2 ± 0.4	3.3 ± 0.4	0.791	0.434
1 d after operation	7.8 ± 0.8	8.2 ± 1.1	2.302	0.027
2 d after operation	6.4 ± 0.7	6.9 ± 0.6	2.425	0.020
3 d after operation	3.6 ± 0.3	4.7 ± 0.5	8.437	<0.001
NSE (*μ*g/L)				
Before operation	5.8 ± 1.2	5.9 ± 0.8	0.310	0.758
1 d after operation	12.3 ± 3.1	14.6 ± 3.4	2.236	0.031
2 d after operation	11.8 ± 2.8	13.7 ± 2.5	2.264	0.029
3 d after operation	6.2 ± 1.6	7.4 ± 1.5	2.447	0.019

The article "Ultrasound Radiomics-Guided Iliac Fascia Block on Postoperative Cognitive Dysfunction in Elderly Patients Undergoing Hip Surgery" was published in 2022. Journal: Comput Math Methods Med.

## Data Availability

The data used to support the findings of this study are available from the corresponding authors upon request.
